# Functional Evaluation of Percutaneous Coronary Intervention Based on CT Images of Three-Dimensional Reconstructed Coronary Artery Model

**DOI:** 10.1155/2023/6761830

**Published:** 2023-04-07

**Authors:** Dongliang Fu, Mengru Liu, Mingjing Shao, Yijin Mao, Chunyan Li, Hong Jiang, Xianlun Li

**Affiliations:** ^1^Department of Cardiology, Integrated Traditional Chinese and Western Medicine, China-Japan Friendship Hospital, No. 2 East Yinghua Road, Chaoyang District, Beijing 100029, China; ^2^Graduate School, Peking Union Medical College, Beijing 100730, China; ^3^Beijing Escope Tech Co Ltd, Beijing, China

## Abstract

In order to explore the computerized tomography (CT) based on three-dimensional reconstruction of coronary artery model, the functional evaluation was made after percutaneous coronary intervention (PCI). In this study, 90 patients with coronary heart disease who received elective PCI were selected. The blood flow reserve fraction (FFR) and SYNTAX score were calculated by three-dimensional reconstruction of CT images, followed up for 2–4 years. According to the SYNTAX score, 0–22 points were defined as the low group (28 cases), 23–32 points as the medium group (33 cases), and 33 points as the high group (29 cases). In this paper, the accuracy, sensitivity, and specificity of CT images of three-dimensional reconstructed coronary artery model are 91%, 73%, and 62%, respectively. The follow-up results showed that the incidence of major adverse cerebrovascular events in the high group was significantly higher than that in the low group and the middle group, and the difference was statistically significant (*P* < 0.05). Pearson correlation analysis showed that SYNTAX score was related to serum total cholesterol (*r* = 0.234, *P*=0.003), triglyceride (*r* = 0.237, *P*=0.014), low-density lipoprotein cholesterol (*r* = 0.285, *P*=0.004), and ApoB/ApoA1 (*R* = 0.004). In this study, FFR is calculated by CT images based on three-dimensional reconstruction of coronary artery model, which can provide support for the diagnosis and treatment of coronary heart disease. SYNTAX score can be used as a risk predictor for PCI patients with coronary heart disease.

## 1. Introduction

Coronary artery heart disease, also known as coronary heart disease, is an ischemic heart disease. It refers to the atherosclerosis of the artery supplying blood to the heart, resulting in lumen stenosis or occlusion, resulting in myocardial ischemia, hypoxia, or necrosis, resulting in chest pain, chest tightness, and other discomfort symptoms [1, 2]. According to *China Cardiovascular Health and Disease Report*, the number of cardiovascular diseases in China has reached 330 million [3]. With the change of people's lifestyle, cardiovascular disease has a younger trend.

With the wide application of percutaneous coronary intervention (PCI) technology, the quality of life of patients with coronary heart disease has been significantly improved [4]. SYNTAX score can reflect the complexity of coronary artery, but with the increase of its value, the incidence of adverse cardiovascular and cerebrovascular events after PCI increases significantly, such as death, stroke, and myocardial infarction [5–7]. Analyzing the influencing factors of SYNTAX score has guiding significance for clinical treatment of coronary heart disease.

At present, the main diagnostic methods of coronary heart disease are coronary angiography and intravascular ultrasound, which is recognized as the “gold standard” of coronary artery diagnosis. However, due to the different degree of coronary artery stenosis, the imaging evaluation is highly subjective, and the influence of the degree of stenosis on the distal blood flow cannot be obtained [8, 9]. In recent years, researchers have used computed tomography (CT) to reconstruct the model of coronary artery in three dimensions and computer blood flow simulation to obtain noninvasive fractional flow reserve (FFR), which has gradually deepened the application of FFR [10]. FFR is defined as the ratio of maximum blood flow at both ends of coronary artery stenosis measured in the case of vascular expansion. When the vessel expands to the maximum, the blood flow of coronary artery is close to the blood pressure value, and the determination of blood pressure value is simpler [11, 12].

In the application process of medical image analysis and processing, medical image segmentation occupies an important position, which not only plays an important role in two-dimensional images, but also attracts much attention in three-dimensional reconstruction. General traditional segmentation of coronary CT image is mainly gray change, edge detection, and only for the ideal image. The emergence of 3D reconstruction technology of medical images has brought important opportunities [13–15]. Three-dimensional reconstruction of medical images can be divided into surface rendering and volume rendering. Surface rendering is widely used because of its simple principle and easy operation. Volume rendering algorithm can see part of the information in the data and provide doctors with clear and reliable internal structure of the organization [16]. Although there are many studies on the evaluation of coronary heart disease based on coronary artery model reconstructed by CT imaging at home and abroad, there is no single method of coronary artery reconstruction.

In this study, according to the existing image segmentation and reconstruction technology, the interactive live wire segmentation based on clustering threshold segmentation was used to segment the coronary artery, and the mobile cube method based on image segmentation was used to reconstruct the three-dimensional CT images of 90 patients with coronary heart disease. Then, the finite element analysis software combined with the method of human hemodynamics was used to analyze the dynamic fluid of the reconstructed model, and the wall pressure of the proximal and distal vessels was obtained, so as to calculate the FFR of the coronary artery. The purpose is to explore the evaluation effect of three-dimensional reconstruction technology based on CT images on coronary heart disease and provide guidance for clinical diagnosis.

## 2. Research Methods

### 2.1. Objects

In this study, 90 patients with coronary heart disease, including 43 males and 47 females, with an average age of (63.35 ± 9.74) years, who were hospitalized from November 20, 2018, to May 20, 2020, and received elective PCI therapy were selected. This study has been approved by ethic committee of the hospital, and patients and their families have signed informed consent.

Inclusion criteria were defined as follows: (1) stable or unstable angina pectoris; (2) stenosis without intervention; (3) at least one of the main epicardial arteries was completely occlusive; (4) left main artery disease accompanied by significant stenosis of other vessels; (5) dysplasia of the right coronary artery; and (6) angiography showed that the diameter of blood vessels was more than 1.5 mm.

Exclusion criteria were defined as follows: (1) accompanied by severe liver insufficiency; (2) accompanied by severe infection and trauma; (3) complicated with malignant tumor; (4) accompanied by severe anemia; and (5) cardiomyopathy, aortic dissection, and congenital heart disease.

### 2.2. Routine Examination

4 mL of venous blood was taken from all patients the next morning after fasting 8 h after admission. Automatic biochemical analyzer was used to detect serum total cholesterol, triglyceride, low-density lipoprotein cholesterol, and other biochemical tests. ApoA1 and ApoB levels were measured by immunoturbidimetry, and ApoB/ApoA1 was calculated. The blood routine, liver and kidney function, blood glucose examination, hypertension, diabetes, smoking history, and other complications were recorded.

### 2.3. CT Coronary Artery Imaging Scanning

64-row definition dual-source CT scanner was used. In supine position, the patient was scanned from 1 cm below the tracheal bifurcation to the diaphragm. The right median cubital vein was punctured with a venous indwelling needle (18 G). 75 mL of iopromide was injected at a rate of 4.5 mL/*s* with a double-tube high pressure syringe, and then saline was injected at a rate of 5 mL/*s*. Tube voltage was 110–130 kV, and tube current was 350–410 mAs. According to the basic heart rate, the acquisition and recombination time window positions were selected. When the heart rate was below 70 times/min, the acquisition phase was (80 ± 9) % R-R interval, and when the heart rate was above 70 times/min, the acquisition phase was (50 ± 9) % R-R interval.

### 2.4. Grouping and Follow-Up Method

All patients completed preoperative examination and underwent CT angiography (CTA) without surgical contraindications. An angiography machine was used to collect images at 25 frames/s and save them by digital subtraction. Left and right coronary angiography was performed by the Seldinger method through femoral artery approach. The contrast agent was 7 mL of iopromide. Multiposition angiography was performed to fully display the main branches and branches of left and right coronary arteries. Combined with the results of angiography, SYNTAX score was calculated according to previous literature. Each vessel with diameter >1.5 mm and stenosis >50% was included in the calculation. In this study, SYNTAX score 0–22 was defined as the low score group (28 cases), 23–32 as the medium score group (33 cases), and 33 as the high score group (29 cases). All 90 patients were followed up by telephone or outpatient.

### 2.5. CT Image Based on 3D Reconstruction of Coronary Artery Model

In this study, since the gray values of each tissue in the coronary CT image are similar and the structure is complex, the clustering threshold segmentation is used to extract similar substances from the image. Firstly, the coronary artery was scanned by the test threshold *t* to create a vector representing the average value. The sum of squares of the difference between each pixel and the average value is calculated, and the calculated sum of squares is the main component of the objective function *G*(*t*). By calculating the value of *G*(*t*) function with all *t*, the minimum *t* corresponding to *G*(*t*) is obtained. The calculation equation is as follows:

(1) $$\begin{array}{c} \bar{a_{1}}=\frac{1}{M_{1}}\sum_{p\in B_{1}}\bar{p}, \end{array}$$

(2) $$\begin{array}{c} \bar{a_{2}}=\frac{1}{M_{2}}\sum_{p\in B_{2}}\bar{p}. \end{array}$$

In equations (1) and (2), $\bar{a_{1}}$ and $\bar{a_{2}}$ represent vectors, M1 and M2 represent the number of pixels in foreground pixels and background pixels, respectively, and *p* represents the vector of pixels. B1 and B2 are the collections of these pixels. The overall average equation is as follows:

(3) $$\begin{array}{c} \bar{a}=\frac{1}{M_{1}+M_{2}}\sum_{p\in B}\bar{p}. \end{array}$$

The basic flow of CT image based on 3D reconstruction of coronary artery model is shown in Figure 1. The CT two-dimensional slice images of patients with coronary heart disease obtained from 64-slice spiral CT scan were stored in CD, and then these CT images were imported into the workstation for classification. After labeling, DICOM images were loaded into the software using 3Dmed. Then, the preprocessing plug-in and image segmentation plug-in were integrated into 3Dmed to segment CT two-dimensional cardiac slice images, extract coronary artery, and construct three-dimensional reconstruction model after registration. Three-dimensional reconstruction based on CT images was implemented in the MITK algorithm library mitkBinMarchingCubes. In addition, the core layer of 3Dmed software calls MITK algorithm library.

### 2.6. Calculation of Coronary FFR

In this study, the ANSYS FLUENT software package is used to analyze the coronary artery fluid dynamics. For the reconstruction of the external model, sometimes it cannot fully meet the model requirements of the finite element analysis. In this study, the Design Modeler in FLUENT must be used to preprocess the three-dimensional reconstruction model before the finite element analysis, so that it can be meshed, laying a good foundation for the later computational fluid dynamics. Because there are many branches of coronary tree and many corresponding outlets, the measurement of flow is limited, and the FFR is calculated according to the pressure value, so the outlet setting conditions are consistent with the pressure conditions. Firstly, the solver is selected to solve the control equation according to the continuous equation, momentum conservation theorem, and fluid equation of energy equation. The calculation equation is as follows:

(4) $$\begin{array}{c} \left(\nabla .v\right)=0, \end{array}$$

(5) $$\begin{array}{c} \rho \frac{dv}{dt}=-\nabla P+\mu \nabla^{2}v. \end{array}$$

In equations (4) and (5), *v* represents velocity vector, *ρ* represents fluid density, *P* represents pressure vector, and *μ* represents fluid viscosity. The pressure value was collected according to the waveform of pressure changing with time, and the FFR was calculated using statistical knowledge. The equation is as follows:

(6) $$\begin{array}{c} FFR=\frac{Ps}{\mathrm{Pr}}. \end{array}$$

In equation (6), Ps represents the mean pressure of the distal coronary artery in the maximum hyperemia state, and Pr represents the mean pressure of the aorta in the maximum hyperemia state.

### 2.7. Statistical Methods

In this study, SPSS 21.0 statistical software was used to analyze the result data. The calculated data conforming to the normal distribution were expressed by the mean standard deviation ($\bar{\text{x}}$ ±*s*), and the *t*-test was used. The calculation data of nonconformity was expressed in percentage (%), which was adopted *χ*^2^ inspection. Pearson correlation analysis was used to analyze the correlation between SYNTAX score and influencing factors. The measurement data were compared among the three groups by analysis of variance. In addition, *P* < 0.05 indicates that the difference is significant.

## 3. Results

### 3.1. Comparison of Clinical Data

Figure 2 shows the comparison of the clinical data of the three groups of patients. Among the 90 patients with coronary heart disease, 16 cases (57.14%) smoked in the low score group, 17 cases (51.52%) in the medium score group, and 14 cases (48.28%) in the high score group. There were 7 cases (25%) of diabetes in the low score group, 6 cases (18.18%) in the middle score group, and 5 cases (17.24%) in the high score group. There were 17 cases (60.71%) of hypertension in the low score group, 18 cases (54.55%) in the medium score group, and 15 cases (55.17%) in the high score group. There were 3 cases of peripheral vascular disease in the three groups. There were 18 cases of hyperlipidemia in the low score group, 16 cases in the medium score group, and 16 cases in the high score group. The comparison of clinical data was not statistically significant (*P* > 0.05).

### 3.2. Results of CT Images Based on Three-Dimensional Reconstruction of Coronary Artery Model

Through the detection data, we found that the accuracy of CTA reconstruction method for measuring FFR was 75%, the accuracy of traditional FFR method was 81%, and the accuracy of CT image three-dimensional reconstruction used in this study was 91%. The sensitivity of CTA reconstruction method was 61%, that of traditional FFR method was 65%, and that of three-dimensional reconstruction of CT image was 73%. The specificity of FFR measured by CTA reconstruction method was 72%, that measured by traditional FFR method was 84%, and that measured by three-dimensional reconstruction of CT image was 62% (Figure 3).

### 3.3. CT Scanning Results

Figure 4 shows CT scanning results of patients with coronary heart disease. Right lung apex solid lesions, irregular shape, the upper layer was dense, and no bronchial gas was equal. A little lower level showed a large range of flake density and ground glass density, a large range of pleural reaction, and edge fuzzy high-density shadow, and there was necrosis area (Figure 4(a)). There was an enlarged lymph node in the vena cava, with calcification in it. The blood vessels near the left aortic arch entered the inferior vena cava downward, and entered the left subclavian vein upward, as shown in Figure 4(b). Right lung mass, double lung inflammation, double lung texture increased, mediastinal point calcification and nodules, aortic and coronary artery wall calcification, pericardial local thickening, and bilateral pleural local was thickened (Figure 4(c)).

### 3.4. Occurrence of Major Adverse Cardiovascular and Cerebrovascular Events

Adverse cardiovascular and cerebrovascular events include stroke, myocardial infarction, and sudden death. During 2–4 years of follow-up, the incidence of major adverse cardiovascular and cerebrovascular events in the high score group was significantly higher than that in the low score group and the medium score group (*P* < 0.05). There was no significant difference in the incidence of major adverse cardiovascular and cerebrovascular events between the low and medium score groups (*P* > 0.05) (Figure 5).

### 3.5. ROC Curve Analysis of the Three Groups of Coronary Stenosis Diagnosed by Three-Dimensional Reconstruction Based on CT Images

The diagnostic area under curve (AUC) of coronary stenosis diagnosed by three-dimensional reconstruction based on CT images had no significant difference (*P* > 0.05). The three groups had high diagnostic accuracy, as shown in Figure 6.

### 3.6. Influencing Factors of SYNTAX Score by Single Factor Analysis of Variance

Pearson correlation analysis was used to analyze the correlation between SYNTAX score and age, gender, serum total cholesterol, triacylglycerol, low-density lipoprotein cholesterol, and ApoB/ApoA1. SYNTAX score and serum total cholesterol (*r* = 0.234, *P*=0.003), triacylglycerol (*r* = 0.237, *P*=0.014), low-density lipoprotein cholesterol (*r* = 0.285, *P*=0.004), ApoB/ApoA1 (*r* = 0.298, *P*=0.017) (Table 1). SYNTAX score single factor analysis of variance of age (*F* = 1.52, *P*=0.625), gender (*F* = 1.85, *P*=0.726), smoking (*F* = 1.26, *P*=0.632), diabetes (*F* = 1.73, *P*=0.245), hypertension (*F* = 0.98, *P*=0.846), hyperlipidemia (*F* = 0.84, *P*=0.718), stable angina pectoris (*F* = 0.97, *P*=0.691), and unstable angina pectoris (*F* = 1.24, *P*=0.812) has no statistical significance on SYNTAX score, as shown in Table 2.

## 4. Discussion

Coronary heart disease is one of the cardiovascular diseases, which has seriously threatened human life and health [17]. On the basis of standardized drug use, PCI has improved the prognosis and quality of life of patients with coronary heart disease to a certain extent. However, 25.3% of patients with coronary heart disease still have major adverse cardiovascular and cerebrovascular events within 1 year after PCI, such as myocardial infarction, stroke, and sudden death. With the deepening of coronary artery complexity, the incidence of major adverse cardiovascular and cerebrovascular events is also increasing [8, 18, 19]. Therefore, the analysis of relevant factors reflecting the complexity of coronary artery is helpful to formulate reasonable intervention measures, which has very important clinical guiding significance.

In this study, CT images of patients with coronary heart disease were collected, and then a three-dimensional reconstruction model based on CT images was constructed to calculate the FFR by solving the pressure value [20]. By comparing the accuracy, sensitivity, and specificity of CTA reconstruction, traditional FFR method, and the three models in this study, the data show that the error caused by calculating the blood flow reserve fraction based on the three-dimensional reconstruction of CT images is lower than that of the other two methods, which has guiding significance for the diagnosis of coronary heart disease.

SYNTAX score is a scoring standard reflecting the complexity of coronary artery disease in coronary artery bypass grafting and PCI for coronary artery stenosis. It is a hierarchical scoring system according to the location, calcification, bifurcation, and severity of coronary artery disease, which can quantitatively evaluate the complexity of coronary artery disease [21, 22]. In this study, SYNTAX score 0–22 was defined as the low score group (28 cases), 23–32 as the medium score group (33 cases), and 33 as the high score group (29 cases). The patients were followed up for 2–4 years after PCI, and the incidence of major adverse cardiovascular and cerebrovascular events in the high score group was significantly higher than that in the low score group and the medium score group (*P* < 0.05). There was no significant difference in the incidence of major adverse cardiovascular and cerebrovascular events between the low and medium score groups (*P* > 0.05). It shows that the incidence of major adverse cardiovascular and cerebrovascular events after PCI is related to the SYNTAX score. Kandzari et al. (2020) [23] reported that the SYNTAX score can predict the incidence of major adverse cardiovascular and cerebrovascular events after PCI, which is consistent with the results of this study.

Pearson correlation analysis showed that SYNTAX score was positively correlated with serum total cholesterol (*r* = 0.234, *P*=0.003), triacylglycerol (*r* = 0.237, *P*=0.014), low-density lipoprotein cholesterol (*r* = 0.285, *P*=0.004), and ApoB/ApoA1 (*r* = 0.298, *P*=0.017). Serum total cholesterol and low-density lipoprotein cholesterol are the indexes reflecting the number of low-density lipoprotein particles. ApoB/ApoA1 is a balance index reflecting antiatherosclerotic lipoprotein and promoting atherosclerosis in the plasma. The larger the value, the more prominent the situation of atherosclerotic lipoprotein in patients with coronary heart disease. The data results show that the coronary artery complexity level is related to the number of low-density lipoprotein particles, which is similar to the results of Fortier et al. (2018) [24].

Single factor analysis of variance showed that age (*F* = 1.52, *P*=0.625), gender (*F* = 1.85, *P*=0.726), smoking (*F* = 1.26, *P*=0.632), diabetes (*F* = 1.73, *P*=0.245), hypertension (*F* = 0.98, *P*=0.846), hyperlipidemia (*F* = 0.84, *P*=0.718), stable angina (*F* = 0.97, *P*=0.691), and unstable angina (*F* = 1.24, *P*=0.812) had no significant effect on SYNTAX score. This shows that the above factors have correlation with the incidence of coronary heart disease, but no significant correlation with the complexity of coronary artery.

## 5. Conclusion

This study constructs a three-dimensional reconstruction model based on CT images to calculate the FFR, which provides support for the diagnosis and treatment of coronary heart disease. SYNTAX score can predict the risk factors of patients with coronary heart disease after PCI. Although this study has completed the goal of calculating the FFR, there are still deficiencies. First, the sample size is small, and it is necessary to expand the sample for prospective research in the later stage. Second, from the final data, there are some errors in the three-dimensional reconstruction model constructed in this study compared with the traditional FFR method, which may be that the factors such as blood gravity and vascular elasticity are not considered. In the later stage, it is necessary to take the relevant physiological factors into consideration for further in-depth study. In conclusion, this study has guiding significance for the prognosis of PCI in the treatment of coronary heart disease.

## Figures and Tables

**Figure 1:** Basic flow of CT image based on three-dimensional reconstruction of coronary artery model.

**Figure 2:** Comparison of clinical data of the three groups. (a) Average age; (b) the sex ratio; (c) proportion of complications; (d) comparison of types of coronary heart disease.

**Figure 3:** 3D reconstruction results of CT images. (a) Comparison of three reconstruction methods; (b) CT image of coronary artery; (c) coronary artery 3D model reconstruction.

**Figure 4:** CT scan results of patients with coronary heart disease. (a) Patient 1, female, 58 years old, presented with left coronary artery stenosis and soft plaque; (b) patient 2, female, 56 years old, presented with calcification and stenosis of anterior descending branch, imbalance between blood supply and myocardial oxygen consumption, resulting in insufficient blood supply; (c) patient 3, male, 61 years old, presented with right coronary artery stenosis.

**Figure 5:** Comparison of main adverse cardiovascular and cerebrovascular events among the three groups.  ^*∗*^Compared with the high score group, *P* < 0.05.

**Figure 6:** ROC curves of the three groups of coronary stenosis based on 3D reconstruction of CT images. (a) Low score group; (b) medium score group; (c) high score group.

**Table 1:** Pearson correlation analysis SYNTAX score.

Index	*r*	95 CI%	*P*
Age	1.262	0.856–1.736	0.214
Gender	1.375	0.752–1.897	0.517
Serum total cholesterol	0.234	0.098–0.426	0.003 ^*∗*^
Triacylglycerol	0.237	0.084–0.529	0.014 ^*∗*^
Low-density lipoprotein cholesterol	0.285	0.095–0.628	0.004 ^*∗*^
ApoB/ApoA1	0.298	0.124–0.135	0.017 ^*∗*^

Note.  ^*∗*^ indicates correlation *P* < 0.05.

**Table 2:** Single factor analysis of variance for SYNTAX score.

Index	*F*	95% CI	*P*
Age	1.52	0.68–1.79	0.625
Gender	1.85	0.85–2.14	0.726
Smoking	1.26	0.87–2.35	0.632
Diabetes	1.73	1.05–2.19	0.245
Hypertension	0.98	0.84–1.52	0.846
Hyperlipidemia	0.84	0.56–1.84	0.718
Stable angina pectoris	0.97	0.63–1.42	0.691
Unstable angina pectoris	1.24	0.87–1.61	0.812

## Data Availability

The data used to support the findings of this study are available from the corresponding author upon request.
